The article "Race, Income, and the Timeliness of Cleft Palate Repair in the United States" was published in 2021. Journal: Cureus.

# Race, Income, and the Timeliness of Cleft Palate Repair in the United States

**DOI:** 10.7759/cureus.13414

**Published:** 2021-02-18

**Authors:** Jennifer L Harb, Kayva L Crawford, Jonathan C Simmonds, Cullen Roberts, Andrew R Scott

**Affiliations:** 1 Otolaryngology - Head and Neck Surgery, Tufts Medical Center, Boston, USA; 2 Otolaryngology - Head and Neck Surgery, University of California San Diego School of Medicine, San Diego, USA; 3 Otolaryngology - Head and Neck Surgery, Massachusetts Eye and Ear, Boston, USA; 4 Surgery, Brigham and Women's Hospital, Harvard Medical School, Boston, USA; 5 Pediatric Otolaryngology and Facial Plastic Surgery, Tufts Children's Hospital, Boston, USA

**Keywords:** race, sex, cleft palate, craniofacial, palatoplasty, economic, disparities, epidemiology, demographics, cleft palate repair

## Abstract

Objective

To determine if differences exist in the timing of cleft palate repair with respect to sex, race, income, and geographical location within the United States.

Design

Retrospective cross-sectional study using the Kids’ Inpatient Database (KID) from 1997 to 2009.

Setting

Inpatient.

Patients

Children with cleft palate with or without cleft lip undergoing inpatient cleft palate repair.

Main outcome measures

Age at the time of palatoplasty (in months) by sex, race, income quartile, and geographic location.

Results

A total of 7,218 children with cleft palate underwent repair at a mean age of 12.1 months (95% CI 12.0-12.3). Females underwent palatoplasty at an older age (13.6 months) than males (13.2 months), a difference of 0.47 months (SE: 0.19, p=0.015). White children underwent surgery at an earlier age (12.1 months) than Black (12.9 months) (difference: 0.73 months, SE: 0.37, p=0.045), Hispanic (12.7 months) (difference: 0.57 months, SE 0.25, p=0.025), and Asian children (15.7 months) (difference: 3.60 months, SE 0.49, p<0.0001). Asian children were also found to undergo repair later than Hispanic (difference 3.03 months, SE 0.51, p<0.0001) and Black (difference: 2.87 months, SE 0.59, p<0.0001) children. Patients born into the highest income brackets were repaired 0.75 months earlier than those in the lowest bracket (SE: 0.26, p=0.005). Patients in the Midwest underwent palatoplasty later (14.3 months) than in the Northeast (12.9 months) (difference: 1.36 months, SE: 0.31, p<0.0001), South (13.2 months) (difference: 1.05 months, SE: 0.36, p=0.004), and West (13.2 months) (difference: 1.09 months, SE: 0.32, p=0.0007).

Conclusions

After controlling for confounding factors, our results suggest that in recent history, Black, Hispanic, and Asian children with cleft palate were repaired later than their White counterparts. In addition, children of affluent families were repaired earliest, and economically disadvantaged children were repaired later than their peers.

The article "Race, Income, and the Timeliness of Cleft Palate Repair in the United States" was published in 2021. Journal: Cureus.

## Introduction

Orofacial clefting, including cleft lip and cleft palate, is the second most common birth defect in the United States after Down Syndrome [1]. In the United States, cleft palate without cleft lip is estimated to occur at a rate of 1:1600 live births [2]. Palatoplasty, or repair of the cleft palate, is a critical procedure for these patients in order to facilitate proper feeding and speech development. The optimal timing of repair has long been debated, as early surgery promotes improved speech outcomes but risks maxillofacial growth impairment.

 The major functional goal of cleft palate repair is to facilitate intelligible speech production [3]. Even after cleft palate repair, a subset of children develop velopharyngeal insufficiency (VPI), allowing air escape into the nasopharynx and impairment of phoneme pronunciation [3]. Rohrich et al. demonstrated that velopharyngeal competence and improved speech outcomes are more common in infants who undergo cleft palate repair before 10.8 months of age [4]. Sullivan et al. similarly demonstrated a 10.2% rate of VPI when patients were repaired at 7-8.9 months, with a near doubling of that rate to 20% among those repaired from 12 to 14.9 months, and 37.8% at >15 months [5].

The benefits of early palatoplasty on VPI rates, however, must be weighed against the potential effect palate surgery can have on maxillary growth. Premature closure of the hard palate has been implicated in restricted maxillary growth, a condition that results in a narrow palatal arch or a hypoplastic maxilla [3]. While the optimal timing of cleft palate repair remains a controversial topic, most centers within the United States favor prioritizing speech outcomes over maxillary growth, as the latter issue may be addressed later in life through orthodontic and maxillofacial interventions available to patients as a routine part of multidisciplinary craniofacial care.

In the United States, healthcare disparities relating to socioeconomic position and race have been well researched and documented in recent years. According to Fiscella et al., these factors are known to affect health care affordability, geographic mobility, access to transportation, education and literacy, and health beliefs, among other metrics [6]. Additionally, it has been established that race and ethnicity are often associated with multiple other dimensions of social disadvantage, including poverty, residential segregation, limited education, unemployment, debt, low health literacy, and limited English proficiency. Greater cumulative social disadvantage is associated with poorer health [7]. Contemporary events have illuminated the need for medical disciplines to examine their role in perpetuating systemic disadvantages for patients of certain socioeconomic or racial sects. In this light, additional studies examining the distribution of healthcare for patients who require palatoplasty is needed.

The article "Race, Income, and the Timeliness of Cleft Palate Repair in the United States" was published in 2021. Journal: Cureus.

Regional variations in the cost of cleft lip and palate surgery have been described previously [2]. Likewise, geographic and socioeconomic differences in the nature and rates of surgical intervention for various craniofacial conditions have also been noted [8]. In 2011, Abbott et al. examined an inpatient pediatric database to identify admissions for cleft palate repair between the years 2003 and 2008 [9]. Their findings suggested that some degree of inequity may exist in regard to the timing of palatoplasty among economically disadvantaged children. The goal of our report is to broaden that previous analysis to over a 12-year period and determine whether race, income percentile, geographic region, or sex significantly impacted the timeliness of cleft palate repair as well. While small differences in the timing of primary palatoplasty may have only minor clinical impact on a child’s overall development, such findings still raise the question of why such discrepancies exist. It is incumbent on cleft surgeons to identify any risk factors for delayed palate repair, which might impart negative effects on speech development. Removing such barriers might mitigate at least one of many factors that potentially compound cultural and economic challenges already present among poor or minority children with cleft palate living in the United States.

## Materials and methods

Data source

A national, de-identified, public database was utilized for this analysis, and institutional review board approval was not required. We utilized the Kids’ Inpatient Database (KID) from 1997 through 2009 to identify patients who were 24 months of age or younger with a diagnosis of cleft palate without cleft lip (ICD 9-CM 749.00-749.04) or cleft palate with cleft lip (ICD 9-CM 749.20-749.25) who underwent primary palatoplasty (ICD-9-CM 27.62). The KID is the only all-payer, pediatric inpatient database in the United States thus the largest centralized source of de-identified patient data. Age in months of the primary repair as well as patient demographic information such as race, sex, location, and income quartile, and hospital region was obtained. Race was defined according to designations established by the KID, including White, Black, Hispanic, Asian or Pacific Islander, Native American, and Other. Patient discharges from 2012 and 2016 were excluded as the KID data entries for these years do not include the age of the patient in months.

The article "Race, Income, and the Timeliness of Cleft Palate Repair in the United States" was published in 2021. Journal: Cureus.

Statistical analysis

Statistical analyses were performed using SAS 9.4 (SAS Institute Inc, Cary, NC). Discharge counts under 11 observations were masked per the HCUP data-use agreement. The data were weighted. A multiple linear regression analysis was performed to control for confounding demographic variables. These variables included race, sex, income quartile, hospital type, and geographic location. The least-square means (LSM) along with the standard error (SE) are reported.

## Results

Between the years 1997 and 2009, 7,218 children with cleft palate underwent surgical repair at a mean age of 12.1 months (95% CI: 12.0-12.3). The mean age at the time of repair for females (13.6 months) was older than males (13.2 months) (difference: 0.47 months, SE: 0.194, p=0.0153) (Table 1).

**Table 1:** LSM age of palatoplasty by sex when controlling for race, hospital location, and socioeconomic status. LSM: least square mean; SE: standard error.

Sex	Age of repair		Difference		
	Months	SE	Months	SE	p-value
Female	13.6	0.40	0.471	0.19	0.02
Male	13.2	0.40			

White children underwent surgery at an earlier age (12.1 months) than Black children (12.9 months) (difference: 0.73 months, SE: 0.37, p=0.045), Hispanic children (12.7 months) (difference: 0.57 months, SE 0.25, p=0.025), and Asian children (15.7 months) (difference: 3.60 months, SE 0.49, p<0.0001) (Table 2).

**Table 2:** LSM age of palatoplasty by race when controlling for sex, hospital location, and socioeconomic status. LSM: least square mean; SE: standard error.

Race	Age of repair	
	Months	SE
Asian	15.7	0.57
Black	12.9	0.46
Hispanic	12.7	0.38
Native American	14.4	1.46
Other	12.6	0.46
White	12.1	0.32

Asian children were also found to undergo repair later than Hispanic children (difference 3.03 months, SE 0.51, p<0.0001) and Black children (difference: 2.87 months, SE 0.59, p<0.0001) (Table 2). The mean age at time of palate repair in the Midwest (14.3 months) was older than children in the Northeast (12.9 months) (difference: 1.36 months, SE: 0.31, p<0.0001), South (13.2 months) (difference: 1.05 months, SE: 0.36, p=0.004), and West (13.2 months) (difference: 1.09 months, SE: 0.32, p=0.0007) (Table 3).

**Table 3:** Comparison of mean age of palatoplasty by hospital region. LSM: least square mean; SE: standard error.

Region	Age of repair	
	Months	SE
Northeast	12.9	0.40
Midwest	14.3	0.47
South	13.2	0.46
West	13.2	0.39

Furthermore, patients born into the lowest income bracket were repaired later (13.7 months) than those born into the highest income bracket (13.0 months) (difference: 0.75 months, SE: 0.26, p=0.005) (Table 4). 

The article "Race, Income, and the Timeliness of Cleft Palate Repair in the United States" was published in 2021. Journal: Cureus.

**Table 4:** Comparison of mean age of palatoplasty by income quartile. LSM: least square mean; SE: standard error.

Socioeconomic Status	Age of repair	
	Months	SE
<25^th^ percentile	13.7	0.41
25^th^ - 50^th^ percentile	13.9	0.42
51^st^ -75^th^ percentile	13.1	0.43
>75^th^ percentile	13.0	0.42

## Discussion

Our results suggest that race and income quartile are closely linked to the timing of cleft palate repair. Specifically, we found that Black, Hispanic, and Asian patients undergo cleft palate repair at significantly older ages than White children (Table 2). We also found that patients with cleft palate born into families in the lowest socioeconomic quartile were consistently repaired later than the mean age of those born into families in the highest income quartile (Table 4).

The results of this analysis are consistent with prior studies of healthcare usage and practices. A study by Fiscella et al. showed that non-White and socioeconomically disadvantaged patients consistently experience delayed treatment and less comprehensive health care, often receiving fewer preventative and routine health measures such as mammograms and immunizations [6]. Differences among races and socioeconomic strata in regards to rates of surgical intervention as well as the timing of such interventions have also been described [2,8]. When examining rates of tongue reduction surgery in children under five years of age with macroglossia, a higher rate of intervention was seen among White children (41.5%) as compared to all other races (27.06%). In addition, a higher rate of tongue reduction was noted in patients within the highest income quartile as compared to all other quartiles (43.29% vs 22.21%) [8]. In the cleft palate literature, Abbott et al. published a study showing that that minority race and public insurance independently predicted later palate repair as compared to White race and private insurance [9]. The mechanisms by which socioeconomic status and race affect access to healthcare are multifactorial, but may include healthcare affordability, access to transportation, geographic location, education, knowledge, literacy, racial concordance between physician and patient, patient attitude and preference, competing demands such as work and childcare, and provider bias among other factors [6].

One of the primary determinants of a successful cleft palate repair is the establishment of velopharyngeal competence, or the convergence of the soft palate against the posterior pharyngeal wall during speech. Children with unrepaired cleft palate show an increased incidence of articulation errors, including non-natural speech productions such as glottal stops, pharyngeal fricatives, and reduced pressure nasalized consonants. In the absence of timely cleft palate repair, compensatory strategies may develop given the need to regulate pressure and airflow in the vocal tract, even at the expense of undermining speech performance. Once learned, compensatory speech patterns are difficult to correct, highlighting the critical role of timely palate repair in optimizing long-term speech outcomes [3]. Numerous studies have suggested that delayed palatoplasty and subsequent VPI lead to adverse physical and psychological sequelae. Delayed palatoplasty has a higher rate of postoperative VPI, with abnormal speech production and reduced intelligibility due to hyper-resonance, audible nasal air emissions, nasal turbulence, and articulation errors [3-5,10-12]. 

The article "Race, Income, and the Timeliness of Cleft Palate Repair in the United States" was published in 2021. Journal: Cureus.

Compounding the effects of abnormal speech among children born with pre-existing societal, economic, and racial disadvantages only serves to reinforce and continue a cycle of inequality in this vulnerable population. Watterson et al. found that a child’s social acceptance by his or her peers decreased as the degree of hypernasality increased and Overby et al. found that teachers expected children with unintelligible speech to struggle more in school, have major literacy delays, and be timid in nature [13,14]. Children and adults with communication disorders are perceived more negatively in terms of intelligence, appearance, behavior, self-esteem, health, competence, social adjustment, education, social appeal, and employability [15].

Several factors may be mitigating the timing of palatoplasty among those patients with the highest family income levels. Rohrich et. al previously demonstrated advantages to performing cleft palate repair prior to 11 months of age in terms of speech outcomes [4,16]. While most authors agree that palatal closure prior to 12 months of age optimizes speech outcomes, it has also been demonstrated that any method of palatoplasty performed prior to the completion of facial growth results in at least some degree of midface hypoplasia [3,4]. It is the responsibility of the surgeon to educate and empower parents to proceed with palatoplasty at an age that will minimize the deleterious effects of maxillary growth restriction without compromising long-term speech outcomes. Armed with this information, it may be that families with robust financial resources and comprehensive medical and dental insurance coverage tend to place less weight on risking maxillofacial growth disturbance in favor of optimizing their child’s speech outcomes.

Among families earning >75th income percentile and White patients, the mean age at palate repair was 13.0 months and 12.1 months, respectively. This observation suggests that these two demographics occupy a position of relative privilege, in which the timing of surgery is consistent with current, evidence-based recommendations in the speech and cleft palate literature. Conversely, our data suggest that cleft palate repair in non-White children takes place weeks to months later than the timeframe that the literature would suggest might optimize speech development.

The article "Race, Income, and the Timeliness of Cleft Palate Repair in the United States" was published in 2021. Journal: Cureus.

We found statistically significant differences in the timing of palatoplasty for females versus males. The reasons for this are not clear but one might postulate that certain factors such as a higher incidence of cleft lip and palate among males and a higher incidence of isolated cleft palate among females may have an unforeseen effect on scheduling palate surgery. For example, infants with isolated cleft palate may be seen at less frequent intervals preoperatively by the cleft surgeon compared to those children who have been followed at more frequent intervals throughout infancy given the additional presence of cleft lip, a defect typically repaired between 3 and 6 months of age. Postoperative visits following lip surgery afford multiple chances for the surgeon and parents to discuss the optimal timing of the next surgery (palatoplasty) and such office visits may also provide families more opportunities to choose a date for palate surgery well ahead of time. Conversely, infants with isolated cleft palate typically require fewer pre-operative visits and their families may therefore have fewer opportunities to take such an active role in scheduling palate surgery months in advance. If this is indeed the reason for such differences in the timing of palate repair, such discrepancies could easily be addressed through protocols that assure a date for cleft palate repair is set for each patient by eight months of age.

Another unexpected finding was that of regional variations in the timing of palatoplasty. Infants in the Midwest tend to undergo palatoplasty later than children in other regions of the United States (Table 3). The reasons for this difference are unclear, and further research is required. One hypothesis for this may be related to a relatively longer travel time from rural and non-urban areas throughout the Midwest to urban treatment centers, some of which are in neighboring states. Access to scheduling, assuring adequate local accommodations for family in the perioperative period, and amassing adequate financial and social resources to allow for a two-to-three-day journey away from home may unknowingly delay surgical dates by a few weeks. Early identification of those patients who will likely incur some degree of social stress or financial hardship in order to make the journey to a regional cleft center for their child’s surgery could allow for a more proactive approach by the craniofacial team. For example, social workers and counselors available for family support could be mobilized early and discussions about the expected dates and length of stay for palate surgery could be initiated earlier in infancy than is typically done to allow for adequate lead time for logistical planning.

The article "Race, Income, and the Timeliness of Cleft Palate Repair in the United States" was published in 2021. Journal: Cureus.

Finally, the late age of repair among Asian children with cleft palate merits comment. This finding is most easily explained by the high rate of adoption of Chinese and South Korean children with craniofacial differences in the United States. In the year 1999, Asian adoptees represented approximately 6% of all adoptive kindergarteners in the United States. By 2011, this percentage had nearly tripled to 17% [17]. When a child with a cleft palate who is living overseas enters adoption proceedings, it is common for the local caregivers to defer further surgical interventions in the child’s native country, with the assumption that delaying such interventions so that they might be performed in the United States is in the best interest of the child. Between the years 2009 and 2011, 49.3% of internationally adopted children under age 6 immigrated from Asia (US Census Bureau, 2009-2011 American Community Survey). It is also noteworthy that a large percentage of Asian adoptions are female, an observation that may also explain the higher mean age of palate repair among females compared to males.

Strengths and limitations

A major strength of this study is the large size and broad range of data comprised in the KID. Using the KID, we were able to analyze a sample size of 7,218 patients who underwent cleft palate repair spanning all regions of the United States over a period of 12 years. This large sample size increases the likelihood that our findings are both valid and generalizable.

The limitations of this study include shortcomings inherent to the KID. As a result of patient deidentification in such a database, we were unable to account for patients who may have had extenuating circumstances that might explain delayed timing of cleft palate repair. One such type of extenuating circumstance that has been touched on above is international adoption. A previous study found that international adoptees with cleft palate were not adopted until a mean age of 22 months and spent seven additional months in the United States prior to cleft palate repair [3]. Since we could not identify international adoptees among the patients in our study, it is not possible to know whether the racial and socioeconomic breakdown of international adoptees skewed the average age at which patients of different sex or racial and socioeconomic groups were repaired.

The article "Race, Income, and the Timeliness of Cleft Palate Repair in the United States" was published in 2021. Journal: Cureus.

This study also did not factor in medical co-morbidities that may have led to delayed repair; given the de-identified nature of the data and the inability to follow an individual patient’s separate hospital admissions over time, it is impossible to parse out these reasons using the KID. An additional limitation is that the KID does not directly provide patient socioeconomic status, and as a result our income classification for patients is an estimate based on the median household income within their family’s zip code. The KID user agreement also does not allow reporting from any group with fewer than 11 patients, which therefore results in the exclusion of some patient groups and possible skewing of the data. However, given that our reported data encompasses a total n of greater than 7,000 patients, it is unlikely that these omissions resulted in a significant data alteration. A final limitation of using the KID is the possibility of inconsistently and potentially inaccurately collected data on patient race. It has been frequently demonstrated that health care entities are inconsistent in the manner in which they determine and collect patient racial data [6,18]. The methods used can vary from patient self-identification to admitting physician observation, and racial categories can vary from a few predefined choices to a “fill in the blank” response [18]. A nationwide sample such as the KID that spans the decades of the 1990s and 2000s undoubtedly includes these and many other methods of categorizing a patient’s race, and our analysis is therefore limited by such inconsistencies.

Finally, we wished to expand the study group to include more recent iterations of the KID including the years 2012 and 2016; however, the data available for those years do not include the age of infants in months, precluding precise analysis of each child’s age at the time of palatoplasty.

## Conclusions

In this large database analysis of 7,218 children undergoing cleft palate repair, we demonstrate that Black, Hispanic, and Asian children with cleft palate undergo palatoplasty later than their White counterparts. Patients in the lowest income quartile are repaired later than children born into more affluent families. Dismissing such observations as mere “minor differences” or “probably clinically insignificant” is missing the point. It is our duty as physicians and providers to identify potential inequities in the delivery of healthcare and correct them. Cleft palate surgeons and those providing care to infants awaiting palatoplasty should be aware of such disparities. Only then can we be proactive in mitigating potential circumstances that contribute to further delays in time-sensitive interventions such as palatoplasty.
